The article "Aircraft Detection for Remote Sensing Image Based on Bidirectional and Dense Feature Fusion" was published in 2021. Journal: Comput Intell Neurosci.

# Aircraft Detection for Remote Sensing Image Based on Bidirectional and Dense Feature Fusion

**DOI:** 10.1155/2021/7618828

**Published:** 2021-09-14

**Authors:** Liming Zhou, Haoxin Yan, Chang Zheng, Xiaohan Rao, Yahui Li, Wencheng Yang, Junfeng Tian, Minghu Fan, Xianyu Zuo

**Affiliations:** ^1^Henan Key Laboratory of Big Data Analysis and Processing, Henan University, Kaifeng, Henan, China; ^2^School of Computer and Information Engineering, Henan University, Kaifeng, Henan, China; ^3^Zhongke Langfang Institute of Spatial Information Applications, Langfang, Hebei, China

## Abstract

Aircraft, as one of the indispensable transport tools, plays an important role in military activities. Therefore, it is a significant task to locate the aircrafts in the remote sensing images. However, the current object detection methods cause a series of problems when applied to the aircraft detection for the remote sensing image, for instance, the problems of low rate of detection accuracy and high rate of missed detection. To address the problems of low rate of detection accuracy and high rate of missed detection, an object detection method for remote sensing image based on bidirectional and dense feature fusion is proposed to detect aircraft targets in sophisticated environments. On the fundamental of the YOLOv3 detection framework, this method adds a feature fusion module to enrich the details of the feature map by mixing the shallow features with the deep features together. Experimental results on the RSOD-DataSet and NWPU-DataSet indicate that the new method raised in the article is capable of improving the problems of low rate of detection accuracy and high rate of missed detection. Meanwhile, the AP for the aircraft increases by 1.57% compared with YOLOv3.

## 1. Introduction

Object detection for remote sensing images, which is considered as the focus issue of remote sensing information processing, exerts an enormous function on aviation and transportation fields. In the wake of developments in the acquisition technology for remote sensing images, we can obtain clearer and higher resolution remote sensing images. These high-resolution images can provide more detailed information, which can help us better identify and locate the corresponding target objects. However, in most cases, the scenario of the aircraft for remote sensing images is usually complex. With the uneven distribution of background and object, the recognition difficulty is easily affected by background noise. What's worse, the object detection algorithm currently in common use for remote sensing image has the problems of low rate of detection accuracy and high rate of missed detection. Therefore, a new method is needed to propose for object detection.

The article "Aircraft Detection for Remote Sensing Image Based on Bidirectional and Dense Feature Fusion" was published in 2021. Journal: Comput Intell Neurosci.

The initial object detection method is generally composed of three parts, and they are region candidate, feature extraction, and classifier classification, respectively. Firstly, the sliding window strategy is used for the candidate regions of interest. Then, features designed manually, such as Haar [1], HOG [2], and DPM [3], are used for withdrawing the candidate regions' features. Finally, classifiers that have been previously trained, such as SVM [4] and Adaboost [5], are utilized for identifying the candidate regions. Traditional methods for object detection, nevertheless, leveraging the strategy of the sliding window for region candidate to improve the area selection strategy. The sliding window strategy is usually blind, needing to design a variety of different window sizes ahead of time. To ensure that objects of different sizes can get candidates, it will produce a great number of redundant candidate windows, leading to the calculation of ascension. In addition, features designed manually usually refer to simple geometric features. Feature extraction based on features designed manually usually does not have robustness for objects in complex scenes and cannot cope well with noise interference caused by the changeable environment.

In the wake of the progress of deep learning, the method on the fundamental of convolutional neural network for object detection has been proposed and widely utilized in a variety of complex scenes. The methods mentioned above are usually composed of two categories, namely, one-stage methods and two-stage methods. One-stage methods, for instance, YOLO [6], SSD [7], and Retinanet [8], distinguish the object detection problem as a classification and regression problem without the need to generate candidate boxes in advance. Instead, images are directly input into the detection network for feature extraction, and then object classification and prediction box regression are carried out simultaneously. Two-stage methods, for instance, R-CNN [9], SPP-NET [10], FAST R-CNN [11], and Faster R-CNN [12], firstly guide the generation of candidate boxes through the predesigned clustering algorithm and then carry out feature extraction operation on the candidate boxes. Then, the classification of the target object and the regression of the prediction box are carried out. One-stage methods, in contrast to the two-stage methods, without the need to generate candidate box area, have much smaller amount of calculation, and the speed is much faster. With the classification and regression carried out simultaneously, it can achieve the training for end-to-end. Although the two-stage methods have lower speeds, with the guidance of the candidate boxes, detection accuracy is higher than the one-stage methods.

The article "Aircraft Detection for Remote Sensing Image Based on Bidirectional and Dense Feature Fusion" was published in 2021. Journal: Comput Intell Neurosci.

A lot of algorithms for aircraft detection have been developed and applied to different scenes. Wang et al. [13] aimed at the problem that there were different scale aircraft objects in the images of remote sensing, establishing a minitype data set and proposing a multiscale aircraft detection algorithm. Hou et al. [14] aimed at the problem that infrared aircraft target was a blur and the detection was easy to be interfered by noise, proposing an improved detection method for microinfrared aircraft target. Zhiyong et al. [15] aimed at the problem that LCCD with VHR optimal images performed poorly because of high intraclass variation and low interclass variance, presenting an overview of the development of LCCD with VHR remote sensing images and discussing the future challenges and opportunities in applying VHR remote sensing images in LCCD. Zhiyong et al. [16] aimed at the problem that existing approaches had limited capability to capture the objects of varying shapes/sizes present in an area impacted by the landslide, developing an algorithm based on automatic adaptive region extension using very-high-resolution remote sensing images. Wang et al. [13] aimed at the problem that spaceborne optical remote sensing images were difficult to obtain and costly, proposing the aircraft detection algorithm which could detect aircraft objects with small samples. Li et al. [17] aimed at detecting the keypoints of aircraft, proposing a category-aware landmark detection network (CALDN) that possessed two streams: a classification stream for size categorization and a localization stream for landmark detection. Zhao et al. [18] aimed at the problem that detecting aircrafts accurately in SAR images was still challenging due to the effects of the special structures of aircrafts and the complexity of SAR imaging mechanism, proposing a novel network called pyramid attention dilated network (PADN). Lin and Chen [19] aimed at the problem that whether directly employing a large number of instances with great variation would lead to a good performance, proposing a you-only-look-once-v3-based detection process for automatic aircraft detection. Yan et al. [20] aimed at the problem that while many advanced works had been developed with powerful learning algorithms in natural images, there still lacked an effective one to detect aircraft precisely in remote sensing images, especially in some complicated conditions, proposing a novel method to detect aircraft precisely, named aircraft detection using Center-based Proposal regions and Invariant Features (CPIF). Wu et al. [21] aimed at the problem that aircraft targets were usually small and the cost of manual annotation was very high, proposing a simple yet efficient aircraft detection algorithm called Weakly Supervised Learning in AlexNet (AlexNet-WSL). Luo et al. [22] aimed at the problem that there were several major challenges in aircraft detection from synthetic aperture radar (SAR) images, such as the shattered features of the aircraft, the size heterogeneity, and the interference of a complex background, proposing an Efficient Bidirectional Path Aggregation Attention Network (EBPA2N). Heiselberg and Heiselberg [23] aimed at the problem that detecting aircrafts in satellite images was a challenge when the background was strongly reflective clouds with varying transparency, proposing a fast and effective detection algorithm that could find almost all aircrafts above and between clouds in Sentinel-2 multispectral images. Shi et al. [24] aimed at the problem that it was still a challenge in remote sensing detection due to complex background and multiscale characteristics, proposing a two-stage aircraft detection method based on deep neural networks, which integrated Deconvolution operation with Position Attention mechanism (DPANet). Xu et al. [25] aimed at the problem that the aircraft to be detected was very small, external environmental factors were easily fused, and the interference of objects to aircraft had a great impact on the aircraft characteristics in remote sensing images, proposing a remote sensing aircraft detection method based on deep learning. Zhou et al. [26] aimed at the problem that the recent algorithms would miss some small-scale aircrafts when applied to the remote sensing image, proposing the Multiscale Detection Network (MSDN), which introduced a multiscale detection architecture to detect small-scale aircrafts. Although lots of methods for aircraft detection have been proposed, there are still many problems when the methods are applied to the remote sensing images, needing a more suitable method for aircraft detection in remote sensing images.

The article "Aircraft Detection for Remote Sensing Image Based on Bidirectional and Dense Feature Fusion" was published in 2021. Journal: Comput Intell Neurosci.

With the intention to address the problem of low rate of detection accuracy and high rate of missed detection, on the fundamental of the object detection algorithm of YOLOv3 [27], this paper analyzes the FPN [28] feature fusion module in YOLOv3 and finds that the feature fusion module only fuses the shallow features. Because shallow features and deep features are not combined effectively, some details will be lost in the process of detection. Therefore, this paper proposes a bidirectional and dense feature fusion detection network. The bidirectional and dense feature fusion detection network fuses the feature map extracted from different detection layers, making the detailed information of the shallow features combined with the semantic information of the deep features, so as to decrease the rate of missed detection and false detection. The main contributions of this paper are as follows:

1. To address the problem of low rate of detection accuracy, this paper proposes the Bidirectional Feature Fusion Detection Network (BFFDN), which not only transmits the shallow layers' detailed information to the deep layers but also transmits the deep layers' semantic information to the shallow layers, making the feature fusion more sufficient and increasing the detection accuracy.
2. To address the problem of the high rate of missed detection, this paper proposes the Dense Feature Fusion Detection Network (DFFDN), which not only shortens the path for feature propagation but also reduces the loss for feature propagation, making full utilized of the features and decreasing the missed detection.
3. To address the problem mentioned above simultaneously, this paper combines the Bidirectional Feature Fusion Detection Network with the Dense Feature Fusion Detection Network and name the novel network structure as the Bidirectional and Dense Feature Fusion Detection Network (BDFFDN), which makes the feature fusion more sufficient and makes fully utilized of the features.

## 2. Related Work

### 2.1. YOLOv3 Detection Framework

The YOLOv3 object detection algorithm adopts Darknet-53 network structure as the backbone network. The backbone network uses the residual connection which is used in the ResNet [29] network for reference, so that the problem of gradient disappearance can be avoided while deepening the network's depth. In order to eliminate the negative effects brought by pooling, a stride of 2 convolutional operations is adopted to replace the pooling operation. The backbone network includes 5 subsampling operations. The input image has to go through 5 subsampling operations when passing through the backbone network, and the output feature image's size becomes 1/32 of the original's. With the intention to enhance the prediction of minitype objects, YOLOv3 uses three different scales of the feature maps for target prediction, and by leveraging the characteristics of the FPN feature fusion for reference, the different scales of the feature maps are spliced together by way of upsampling. The YOLOv3 network structure is shown in Figure 1. As we can clearly catch from the figure, if the size of the input image is 416 × 416, the backbone network gets Predict1 at the 82nd Layer after convolution of several layers, that is, the 13 × 13 detection scale. The feature map at the 82nd Layer gets 32 times subsampling operation, and the feature map is appropriate for detecting max-type objects due to the large scale receptive field it has. The backbone network performs an upsampling operation on the 79th layer's feature map and performs feature fusion with the 61st layer's feature map to obtain the feature map at the 91st layer. The backbone network gets Predict2 at the 94th Layer after convolution of several layers, that is, the 26 × 26 detection scale. The feature map at the 94th Layer gets 16 times subsampling operation, and the feature map is appropriate for detecting middle-type objects due to the middle scale receptive field it has. The backbone network performs an upsampling operation on the 91st layer's feature map and performs feature fusion with the 36th layer's feature map to obtain the feature map at the 103rd layer. The backbone network gets Predict3 at the 106th Layer after convolution of several layers, that is, the 52 × 52 detection scale. The feature map at the 106th Layer gets 8 times subsampling operation, and the feature map is appropriate for detecting minitype objects due to the small-scale receptive field it has.

The article "Aircraft Detection for Remote Sensing Image Based on Bidirectional and Dense Feature Fusion" was published in 2021. Journal: Comput Intell Neurosci.

The prediction of the boundary box is shown in Figure 2, where the dark blue box stands for the predicted boundary box and the light blue box stands for the prior box. The purpose of the prediction of the boundary box is to forecast the boundary box's position through the prior box so that the predicted position of the boundary box is closer to that of the real box. The prediction formulas of the boundary box are shown in the following equations:

(1) $$\begin{array}{c} b_{x}=\sigma \left(t_{x}\right)+c_{x}, \end{array}$$

(2) $$\begin{array}{c} b_{y}=\sigma \left(t_{y}\right)+c_{y}, \end{array}$$

(3) $$\begin{array}{c} b_{w}=p_{w}e^{t_{w}}, \end{array}$$

(4) $$\begin{array}{c} b_{h}=p_{h}e^{t_{h}}, \end{array}$$

where *t*_*x*_, *t*_*y*_ represent the center point's coordinates of the prediction box relative to the center point of the cell, *t*_*w*_, *t*_*h*_ represent the prediction box's length and width relative to the prior box, *σ* represents the sigmoid activation function, *σ*(*t*_*x*_), *σ*(*t*_*y*_) represent the offset based on the upper-left coordinates of the center point of the rectangle, *p*_*w*_, *p*_*h*_ represent the length and width of the corresponding a priori box, *c*_*x*_, *c*_*y*_ represents the coordinates of the upper-left corner of the cell, and *b*_*x*_, *b*_*y*_, *b*_*w*_, *b*_*h*_ stand for the prediction box's position and the length and the width.

The loss of YOLOv3 is composed of three parts: coordinate loss, confidence loss, and category loss. The formula of coordinate loss, confidence loss, and category loss is shown in the following equations, respectively:

(5) $$\begin{array}{c} lbox=\lambda_{coor\;d}\overset{S^{2}}{\underset{i=0}{\sum }}\overset{B}{\underset{j=0}{\sum }}l_{i,j}^{obj}\left(2-w_{i}*h_{i}\right)\left[{\left(x_{i}-{\hat{x}}_{i}\right)}^{2}+{\left(y_{i}-{\hat{y}}_{i}\right)}^{2}+{\left(w_{i}-{\hat{w}}_{i}\right)}^{2}+{\left(h_{i}-{\hat{h}}_{i}\right)}^{2}\right], \end{array}$$

(6) $$\begin{array}{c} \text{lobj}=\lambda_{\text{noobj}}\overset{S^{2}}{\underset{i=0}{\sum }}\sum_{j=0}^{B}l_{i,j}^{\text{noobj}}{\left(c_{i}-{\hat{c}}_{i}\right)}^{2}+\lambda_{\text{obj}}\overset{S^{2}}{\underset{i=0}{\sum }}\overset{B}{\underset{j=0}{\sum }}l_{i,j}^{\text{obj}}{\left(c_{i}-{\hat{c}}_{i}\right)}^{2}, \end{array}$$

(7) $$\begin{array}{c} \text{lcls}=\lambda_{\text{class}}\overset{S^{2}}{\underset{i=0}{\sum }}\overset{B}{\underset{j=0}{\sum }}l_{i,j}^{\text{obj}}\underset{c\in \text{classes}}{\sum }p_{i}\left(c\right)\log\left({\hat{p}}_{i}\left(c\right)\right), \end{array}$$

where *λ*_coord_ stands for the weight of coordinate error, *λ*_noobj_ represents the weight of no-target error, *λ*_obj_ represents the weight of target error, *λ*_class_ represents the weight of the classification error; where S represents the grid size, for the 416 × 416 images, the three grid sizes are 13,26 and 52, respectively; where **B** stands for the bounding boxes' number, *l*_*i*,*j*_^obj^ stands for if there is a target object in the bounding box at the *j* position of the *i* grid, if there is a target object, then the value of *l*_*i*,*j*_^obj^ is 1, otherwise is 0. As well, *l*_*i*,*j*_^noobj^ represents if there is not a target object in the bounding box at the *j* position of the *i* grid. If there is not a target object, then the value of *l*_*i*,*j*_^noobj^ is 1, otherwise is 0, where *x*, *y*, **w**, *h*, *c*, *p*(*c*) stands for the true box's center coordinates, width, height, confidence, and probability of the category, respectively, $\hat{x}$, $\hat{y}$, $\hat{w}$, $\hat{h}$, $\hat{c}$, $\hat{p}\left(c\right)$ represent the bounding box's center coordinates, width, height, confidence, and probability of the category, respectively, where 2 − *w∗h* represents the scale factor, the smaller the target object is, the larger the regression loss is, and the stronger the detection effort for detection the small objects.

The article "Aircraft Detection for Remote Sensing Image Based on Bidirectional and Dense Feature Fusion" was published in 2021. Journal: Comput Intell Neurosci.

### 2.2. FPN Feature Fusion Module

Because the shallow layers' features include more detailed information, and the deep layers' features include more semantic information. With the process of downsampling constantly, the feature map will contain more and more semantic information while with less and less detailed information. However, most object detection algorithms focus on the deep layers' features only and ignore the shallow layers' features, leading to inaccurate target positioning.

To settle the problem down, the FPN Feature Fusion Module is proposed. The FPN Feature Fusion Module is capable of integrating the shallow layers' features with the deep layers' features by introducing the feature pyramid structure, making the fused feature map have both the shallow layers' detailed information and the deep layers' semantic information. The FPN Feature Fusion Module is shown in Figure 3, in which the operation downsampling × 0.5 represents 2 times downsampling, Conv1, Conv2, Conv3 represents the 2 times, 4 times, and 8 times downsampling, respectively, the operation 1 × 1 represents using the 1 × 1 convolution size to adjust the number of channels, the operation 3 × 3 represents using the 3 × 3 convolution size to eliminate the effect of confusion by upsampling, and the operation upsampling × 2 represents the 2 times upsampling. Mix2 is formed by feature splicing of Mix3 after 2 times upsampling with Conv2 after 4 times downsampling, and Mix1 is formed by feature splicing of Mix2 after 2 times upsampling with Conv1 after 2 times downsampling. In this way, the spliced Mix1 and Mix2 not only contain more detailed information from the shallow layers but also contain more semantic information from the deep layers, and then use three feature maps of different scales, namely, Mix1, Mix2, and Mix3, to make predictions.

## 3. Proposed Method

### 3.1. Bidirectional Feature Fusion Module

FPN Feature Fusion Module transmits the shallow features' detailed information to the deep features by means of upsampling, so that deep features have the shallow features' detailed information. However, it does not transfer the deep features' semantic information to the shallow features, so that the feature fusion is not sufficient. With the intention to let the shallow features have the deep features' semantic information, this paper proposes the Bidirectional Feature Fusion Module. The Bidirectional Feature Fusion Module is shown in Figure 4. The Bidirectional Feature Fusion Module, based on the FPN Feature Fusion Module, not only passes the feature of Mix3 to Conv2 by upsampling to form Mix2 and passes the feature of Mix2 to Conv1 by upsampling to form Mix1 but also makes the feature splice of Mix1′ after 2 times downsampling with Mix2 to from Mix2′ and makes the feature splice of Mix2′ after 2 times downsampling with Mix3 to form Mix3′, and then using three different scales of feature maps, namely Mix1′, Mix2′, and Mix3′, to make predictions. This paper introduces the Bidirectional Feature Fusion Module into the YOLOv3 method and names the new method Bidirectional Feature Fusion Detection Network (BFFDN).

The article "Aircraft Detection for Remote Sensing Image Based on Bidirectional and Dense Feature Fusion" was published in 2021. Journal: Comput Intell Neurosci.

### 3.2. Dense Feature Fusion Module

The FPN Feature Fusion Module transmits the shallow features' detailed information to the deep features by way of upsampling so that the deep features have the shallow features' detailed information. However, in the process of feature transmission, some features and details will be lost due to the upsampling operation for several times. With the intention to reduce the loss of features, the Dense Feature Fusion Module is proposed through the study of DenseNet [30]. The Dense Feature Fusion Module is shown in Figure 5. The Dense Feature Fusion Module, based on the FPN Feature Fusion Module, not only passes the feature of Mix3 to Conv2 by upsampling to form Mix2 and passes the feature of Mix2 to Conv1 by upsampling to form Mix1 but also makes the feature splice of Mix3 after 4 times upsampling with Conv1 and transmits the feature information of Mix3 directly to Conv1. The operation shortens the transfer path from Mix3 to Mix2 to Mix1 so that the feature loss caused by multiple times upsampling is alleviated and the feature information of Mix1 is enriched and then, using three different scales of feature maps, namely Mix1, Mix2, and Mix3, to make predictions. This paper introduces the Dense Feature Fusion Module into the YOLOv3 method and names the new method Dense Feature Fusion Detection Network (DFFDN).

### 3.3. Bidirectional and Dense Feature Fusion Module

To make the feature map have the shallow features' detailed information and the deep features' semantic information and shorten the path of feature propagation, this paper combines the Bidirectional Feature Fusion Module with the Dense Feature Fusion Module and formats the Bidirectional and Dense Feature Fusion Module. The Bidirectional and Dense Feature Fusion Module is shown in Figure 6. The Bidirectional and Dense Feature Fusion Module has the advantages of the Bidirectional Feature Fusion Module and the Dense Feature Fusion Module, making feature splice of Mix3 after 2 times upsampling with Conv2 and making feature splice of Mix3 after 4 times upsampling with Conv1, making splice of Mix2 after 2 times upsampling with Conv1, making feature splice of Mix1′ after 2 times downsampling with Mix2 and making feature splice of Mix1′ after 4 times downsampling with Mix3, and making feature splice Mix2′ after 2 times downsampling with Mix3, and then using three different scales of feature maps, namely Mix1′, Mix2′, and Mix3′, to make predictions. This paper introduces the Bidirectional and Dense Feature Fusion Module into the YOLOv3 method and names the new method Bidirectional and Dense Feature Fusion Detection Network (BDFFDN).

The article "Aircraft Detection for Remote Sensing Image Based on Bidirectional and Dense Feature Fusion" was published in 2021. Journal: Comput Intell Neurosci.

## 4. Experiments' Results and Analysis

### 4.1. Experimental Environments

The operating system used in this paper is Ubuntu16.4.0, the processor is Intel(R) Xeon(R) Silver 4114 CPU @ 2.20 GHz, and the graphics card is two-piece Quadro P4000. The dataset adopted is the RSOD-DataSet annotated by Wuhan University [31, 32]. Some examples of the RSOD-DataSet are shown in Figure 7. RSOD includes four kinds of objects, including aircraft, oil tank, playground, and overpass and contains a total of 976 pictures, each of which is about 1100 × 900 pixels in size. And the aircraft contains 446 pictures with a total of 4,993 targets, the oil tank contains 165 pictures with a total of 1,586 targets, the playground contains 189 pictures with a total of 191 targets, and the overpass contains 176 pictures with a total of 180 targets. The annotation format of the RSOD is the VOC format, and the annotation is saved in the XML file. Each picture corresponds to an XML file, which contains the target object's position and scale. The position of the target object is represented by the coordinates of the top left corner and the bottom right corner. The ratio of the training set to the test set is 4 to 1. For the aircraft target, the train set contains 356 pictures and the test set contains 90 pictures. In the experiment, learning rate attenuation is adopted to adjust the learning rate. The initial learning rate is 0.001, momentum is 0.9, weight attenuation is 0.0005, and the number of iterations is 40200. As the iterations reach the 32000 generations and 36000 generations, respectively, the learning rate is adjusted to 0.1 and 0.01 of the initial learning rate, respectively. In this way, the convergence speed of loss can be adjusted.

### 4.2. Experimental Results

Loss curve is one of the performance indicators to evaluate the object detection algorithm. Generally speaking, the smaller the loss value of a model is, the better the model is trained and the better the training effect will be. The loss comparison of different models is shown in Figure 8, where the horizontal axis stands for the loss value and the vertical axis stands for the iteration number. It can be clearly seen from the figure that the loss value of different models decreases rapidly between 0 and 2000 iterations. After 3000 iterations, the loss value of different models gradually tends to be stable and fluctuates within a certain small range. Between 35000 and 40200 iterations, it can be seen that the BDFFDN algorithm is at the lowest point of loss value, which means that compared with the YOLOv3 algorithm, BFFDN algorithm, and DFFDN algorithm, the BDFFDN algorithm has a better training effect.

The article "Aircraft Detection for Remote Sensing Image Based on Bidirectional and Dense Feature Fusion" was published in 2021. Journal: Comput Intell Neurosci.

IOU Curve is one of the performance indicators to evaluate the object detection algorithm. IOU stands for the overlapping area between the predicted boundary box and the labeled real box, that is, the ratio of their intersection and union. The closer the value is to 1, the greater the overlap area between the predicted bounding box and the labeled real box will be, and the closer the predicted bounding box is to the labeled real box. The calculation formula of IOU is shown in the following equation:

(8) $$\begin{array}{c} \text{IOU}=\frac{\text{Predict}\cap \text{GroundTruth}}{\text{Predict}\cup \text{GroundTruth}}, \end{array}$$

where Predict represents the predicted bounding box calculated by the network model, GroundTruth represents the labeled real box. The IOU curve comparison of different models is shown in Figure 9, where the horizontal axis represents the IOU value, and the vertical axis represents the iteration number. As can be seen from the figure, the IOU value fluctuates greatly at the beginning of training. As the number of iterations increases, the value of IOU gradually tends to be stable and fluctuates within a certain range. Compared with the YOLOv3 algorithm, BFFDN algorithm and DFFDN algorithm, the fluctuation of IOU of the BDFFDN algorithm is smaller and tends to 0.8.

The P-R Curve comparison of different models is shown in Figure 10, where the horizontal axis represents the Precision, and the vertical axis represents the Recall. The area of the P-R curve represents the performance of the model. Generally speaking, the larger the area of the P-R curve is, the better the performance of the model is. It can be clearly seen from the figure that the YOLOv3 algorithm occupies the smallest area compared with other algorithms, followed by the BFFDN algorithm, followed by the DFFDN algorithm, and finally BDFFDN algorithm. BDFFDN algorithm occupies the largest area compared with other algorithms, which means that the BDFFDN algorithm has the best performance.

In addition to Precision, Recall, IOU, and other performance indicators, *F*1-ccore, AP, and FPS can also be used as indicators to evaluate object detection algorithms. For aircraft object detection, the positive example is aircraft, and the negative example is the objects other than aircraft. Generally, we call the correctly classified positive examples TP, the misclassified positive examples FP, the correctly classified negative examples TN, and the misclassified negative examples FN. For the RSOD-DataSet, the aircraft contains 446 images and a total of 4993 targets. The train set and the test set are divided according to the ratio of 4 to 1. The performance indicators of the aircraft test set are shown in Table 1. For the YOLOv3 algorithm, TP = 936, FP = 99, FN = 116, for the BFFDN algorithm, TP = 990, FP = 44, FN = 62, for the DFFDN algorithm, TP = 998, FP = 33, FN = 54, and for the BDFFDN algorithm, TP = 997, FP = 28, FN = 55. It can be clearly seen from the table that the performance of the BDFFDN algorithm is higher than that of other algorithms, and the visualization of the performance indicator comparison chart is shown in Figure 11. The calculation formulas of performance indexes of Precision, Recall, F1-Score, and AP are shown in the following equations, respectively:

(9) $$\begin{array}{c} \text{Precision}=\frac{\text{TP}}{\text{TP}+\text{FP}}, \end{array}$$

(10) $$\begin{array}{c} \text{Recall}=\frac{\text{TP}}{\text{TP}+\text{FN}}, \end{array}$$

(11) $$\begin{array}{c} F1-\text{Score}=2*\frac{\text{Precision}*\text{Recall}}{\text{Precision}+\text{Recall}}, \end{array}$$

(12) $$\begin{array}{c} \text{AP}=\int_{0}^{1}\text{Precision}\left(\text{Recall}\right)d\text{Recall}. \end{array}$$

The contrastive results in the RSOD-DataSet are presented in Table 2. From Table 2, we are capable of seeing that the mAP of BDFFDN is 91.41%, which increases by 18.44%, 16.34%, 15.55%, 15.43%, 14.83%, 13.62%, 3.65%, 3.49%, 3.08%, 2.68%, and 1.99% compared with SSD, DSSD, FFSSD, ESSD, DC-SPP-YOLO, UAV-YOLO, FRCN, DConvNet, MRFF-YOLO, Improved-YOLOv3, and SigNMS, respectively. The results demonstrate that our proposed method has superior performance than other algorithms. Although the index of FPS is not very high compared with other algorithms and the AP for overpass is not the highest among the algorithms, it could still meet the basic demand for aircraft detection.

The article "Aircraft Detection for Remote Sensing Image Based on Bidirectional and Dense Feature Fusion" was published in 2021. Journal: Comput Intell Neurosci.

As shown in Figure 12, there are 20 images for comparing the detection result of YOLOv3 with BDFFDN. Among these images, the 1st column and the 2nd column are the detection result of YOLOv3, and the 3rd column and the 4th column are the detection result of BDFFDN. From Figure 12, we can clearly see that the objects in the images are mostly in small size, and the objects are distributed densely, which increases the difficulty of detection. The detection result of YOLOv3 has shown the result that YOLOv3 has defectiveness when detecting the small-size objects and missing the small-size objects, while our proposed method has detected the objects missed by YOLOv3. This demonstrates that our proposed method, BDFFDN, has better performance when detecting the small-size objects for remote sensing images than YOLOv3.

### 4.3. Extended Experiments

With the intention to prove the algorithm's generality and generalization, besides the experiments in the RSOD-DataSet, we also do the experiments in the NWPU-DataSet. The NWPU-DataSet [42–44] is a remote sensing dataset used for object detection, which consists of ten kinds of objects, including airplane, ship, storage tank, baseball diamond, tennis court, basketball court, ground track field, harbor, bridge, and vehicle. It contains a total of 800 pictures, of which 650 pictures were used for the positive image set and 150 pictures used for the negative image set. The ratio of the training set to test set is 4 to 1. The total number of iterations is 40200 generations, the learning rate is initialized to 0.001, and the method of constant attenuation is adopted. As the iterations reach the 32000 generations, the learning rate is 0.0001, and as the iterations reach the 36000 generations, the learning rate is 0.00001.

The contrastive results in the NWPU-DataSet are presented in Table 3. From Table 3, we are capable of seeing that the mAP of BDFFDN is 88.99%, which increases by 43.08%, 24.88%, 21.49%, 16.36%, 12.59%, 12.49%, 11.49%, 9.89%, 6.39% compared with EB-V-F-BR, AD-FCN, CPISNet^*∗*^, RICNN, FRCN, R-P-FRCN, NEOON, DConvNet, and DNN, respectively. The results demonstrate that our proposed method has superior performance than other algorithms. Although the AP for ship, storage tank, baseball diamond, basketball court, and vehicle is not the highest among the algorithms, it could still be acceptable.

As shown in Figure 13, there are 20 images for comparing the detection result of YOLOv3 with BDFFDN. Among these images, the 1st column and the 2nd column are the detection result of YOLOv3, and the 3rd column and the 4th column are the detection result of BDFFDN. Through the comparison of the detection result, we are capable of seeing that our method has detected the objects YOLOv3 missed, which demonstrates our method has superior performance than YOLOv3.

## 5. Conclusions

This paper focuses on the issues of low rate of detection accuracy and high rate of missed detection and finds that the FPN Feature Fusion Module has the problem of insufficient fusion of shallow layers and deep layers through the research of the FPN Feature Fusion Module, which will lead to an insufficient combination of the shallow features' detailed information and the deep features' semantic information, and thus lead to inaccurate positioning of small targets, proposing the Bidirectional and Dense Feature Fusion Detection Network and carrying out the experiments on the RSOD-DataSet and NWPU-DataSet. Experimental data show that the proposed Bidirectional and Dense Feature Fusion Detection Network is significantly better than the YOLOv3 object detection algorithm in Precision, Recall, *F*1-score, IOU, AP, and other performance indicators, and detects various small targets that YOLOv3 object detection algorithm cannot detect. With the increase of the detection accuracy and the decrease of missed detection, the computation cost of the method has increased and the detection speed has decreased. In the future direction, how to decrease the computation cost while increasing the detection accuracy will be researched.

The article "Aircraft Detection for Remote Sensing Image Based on Bidirectional and Dense Feature Fusion" was published in 2021. Journal: Comput Intell Neurosci.

## Figures and Tables

**Figure 1:** YOLOv3 network structure.

**Figure 2:** Bounding box prediction.

**Figure 3:** FPN feature fusion module.

**Figure 4:** Bidirectional feature fusion module.

**Figure 5:** Dense feature fusion module.

**Figure 6:** Bidirectional and dense feature fusion module.

**Figure 7:** Some examples of the RSOD-DataSet. (a, b) Aircraft targets; (c, d) oil tank targets; (e, f) playground targets; (g, h) overpass targets.

**Figure 8:** The loss comparison of different models.

**Figure 9:** The IOU curve comparison of different models.

**Figure 10:** The P-R curve comparison of different models.

**Figure 11:** The visualization of performance indicator comparison chart.

**Figure 12:** The comparison results of YOLOv3 and BDFFDN in the RSOD-DataSet. (a1–a10) the detection results of YOLOv3; (b1–b10) the detection results of BDFFDN.

**Figure 13:** The comparison results of YOLOv3 and BDFFDN in the NWPU-DataSet. (a1–a10) the detection results of YOLOv3; (b1–b10) the detection results of BDFFDN.

**Table 1:** The performance indicators of the aircraft test set.

	TP	FP	FN	Precision (%)	Recall (%)	*F*1-ccore (%)	IOU (%)	AP (%)	FPS
YOLOv3	936	99	116	90.43	88.97	89.70	67.42	89.24	**30**
BFFDN	990	44	62	95.74	94.11	94.92	75.68	90.21	28
DFFDN	998	33	54	96.80	**94.87**	95.82	76.00	90.77	28
BDFFDN	**997**	**28**	**55**	**97.27**	94.77	**96.00**	**78.59**	**90.81**	26

**Table 2:** The contrastive results in the RSOD-DataSet.

Method	Backbone	AP (%)					FPS
		Aircraft	Oil tank	Overpass	Playground	mAP	
SSD [7]	VGG-16	69.17	71.20	70.23	81.26	72.97	**61.5**
DSSD [33]	ResNet-101	72.12	72.49	72.10	83.56	75.07	6.1
FFSSD [34]	VGG-16	72.95	73.24	73.17	84.08	75.86	38.2
ESSD [35]	VGG-16	73.08	72.94	73.61	84.27	75.98	37.3
DC-SPP-YOLO [36]	Figure 5 in [35]	73.16	73.52	74.82	84.82	76.58	33.5
UAV-YOLO [37]	Figure 1 in [36]	74.68	74.20	76.32	85.96	77.79	30.12
FRCN [12]	VGG-16	85.85	86.67	88.15	90.35	87.76	6.1
DConvNet [38]	ResNet-101	71.87	90.35	**89.59**	99.88	87.92	6.7
MRFF-YOLO [39]	Figure 5 in [38]	87.16	86.56	87.56	92.05	88.33	25.1
Improved-YOLOv3 [40]	Figure 3 in [39]	86.42	87.57	89.37	91.56	88.73	25.8
SigNMS [41]	VGG-16	80.60	90.60	87.40	99.10	89.40	6.7
BDFFDN (ours)	Figure 6	**90.81**	**90.73**	84.12	**100.00**	**91.41**	26

The article "Aircraft Detection for Remote Sensing Image Based on Bidirectional and Dense Feature Fusion" was published in 2021. Journal: Comput Intell Neurosci.

**Table 3:** The contrastive results in the NWPU-DataSet.

AP (%)	Method									
	EB-V-F-BR [45]	AD-FCN [46]	CPISNet^*∗*^ [47]	RICNN [44]	FRCN [12]	R-P-F RCN [48]	NEOON [49]	DConvNet [37]	DNN [50]	BDFFDN (ours)
Airplane	47.85	69.38	43.10	88.35	82.80	90.40	78.29	87.30	92.40	**99.02**
Ship	35.41	61.82	58.20	77.34	77.50	75.00	**81.68**	81.40	79.30	78.89
Storage tank	63.52	69.66	74.60	85.27	52.50	44.40	**94.62**	63.60	87.10	90.67
Baseball diamond	42.91	62.58	86.20	88.12	**96.30**	89.90	89.74	90.40	93.20	90.68
Tennis court	52.47	61.23	74.50	40.83	62.90	79.70	61.25	81.60	81.00	**90.91**
Basketball court	55.57	73.21	83.60	58.45	68.80	77.60	65.04	74.10	**89.30**	81.50
Ground track field	47.47	75.28	92.50	86.73	98.40	87.70	93.23	90.30	75.80	**100.00**
Harbor	39.85	57.83	66.60	68.60	82.50	79.10	73.15	75.30	72.50	**90.70**
Bridge	36.83	53.77	35.70	61.51	78.80	68.20	59.46	71.40	72.80	**86.23**
Vehicle	37.26	56.38	59.70	71.10	63.80	73.20	78.26	75.50	**83.00**	81.30
mAP	45.91	64.11	67.50	72.63	76.40	76.50	77.50	79.10	82.60	**88.99**

## Data Availability

The research data come from the network public data sets.
